The article "An Insight on the Maternal-Fetal Outcomes of Critically Ill Pregnant Women During the Second Wave of COVID-19" was published in 2022. Journal: Cureus.

# An Insight on the Maternal-Fetal Outcomes of Critically Ill Pregnant Women During the Second Wave of COVID-19

**DOI:** 10.7759/cureus.20998

**Published:** 2022-01-06

**Authors:** Saima Faraz, Nighat Aftab, Abeer Ammar, Israa Al Mulai, Litty Paulose, Shalini Fernandes

**Affiliations:** 1 Obstetrics and Gynecology, Dubai Medical College, Dubai, ARE; 2 Obstetrics and Gynecology, Latifa Women and Children Hospital, Dubai, ARE

**Keywords:** perinatal care, postpartum period, peripartum period, pregnant women, covid-19, critical illness

## Abstract

Background: Coronavirus disease 2019 (COVID-19) and other respiratory infections have been attributed to causing severe disease and pneumonia in pregnant women because of physiological stress and alterations in the immune system during pregnancy. Pregnant women are prone to develop serious outcomes for both mother and child when infected by previous coronaviruses, but there is a paucity of data regarding clinical characteristics and maternal-fetal outcomes in COVID-19. Moreover, various laboratory and radiological parameters are scarcely studied in pregnant women in the third trimester who develop severe COVID-19. Therefore, we conducted this study to assess and compare the maternal-fetal outcomes of critically ill pregnant women with COVID-19 pneumonia who required admission to the intensive care unit (ICU).

Materials and methods: We conducted this retrospective observational study at a tertiary care hospital affiliated with an academic center in the United Arab Emirates. A total of 123 patients in their third trimester were included in the study from December 1, 2020, to March 31, 2021, comprising 30 cases of severe or critical COVID-19 and 93 mild to moderate COVID-19 patients. We collected and analyzed maternal demographic data and radiological and biochemical profiles. We also compared maternal-fetal outcomes.

Results: Thirty patients (24.3%) were admitted to the ICU, and eight required invasive ventilation. Severe COVID-19 pneumonia was significantly associated with higher mortality (20% vs. 0%; p < 0.001), postpartum complications (50% vs. 9.67%; p < 0.001), and increased overall hospital stay than mild to moderate COVID-19 (p < 0.001). In addition, the primary indication for intervention in severe cases was worsening of COVID-19 pneumonia, and pregnant patients had significantly greater chances of undergoing delivery by Cesarean section (80% vs. 40.8%; p = 0.01). Neonates born to severe COVID-19 patients had significantly higher chances of being born preterm (76.6% vs. 35.7%; p < 0.001) and had low birth weight (46.6% vs. 13.9%; p-value = 0.002). There were four stillbirth cases, two vertical transmission cases, and no neonatal deaths.

Conclusions: This study assessed and compared maternal-fetal outcomes of critically ill pregnant women with COVID-19 pneumonia who required admission to the ICU because of the paucity of data in this patient demographic. Pregnant women with severe COVID-19 have high mortality, peripartum complications, increased hospital stay, and are more likely to undergo Cesarean section delivery because of COVID-19 progression than pregnant patients with less severe forms of COVID-19. The newborns born to such mothers may be premature and have low birth weights but have similar mortality to those born to mothers with mild to moderate COVID-19.

## Introduction

Coronavirus disease 2019 (COVID-19) is speculated to be a zoonotic disease that was first reported in the Wuhan province of China in December 2019 and caused by the severe acute respiratory syndrome coronavirus 2 (SARS-CoV-2) [1-2]. COVID-19 and other respiratory infections have been attributed to causing severe disease and pneumonia in pregnant women because of physiological stress and alterations in the immune system during pregnancy [3]. In the past coronavirus outbreaks, it was evident that pregnant women are prone to develop serious outcomes for both mother and child as admission to intensive care units (ICUs), invasive ventilation, miscarriage, preterm delivery, stillbirths, low birth weight, and organ failure and reported mortality was as high as 10% in some case series [4-5].

There is a paucity of data regarding clinical characteristics and maternal-fetal outcomes in COVID-19. The first study to evaluate pregnant women with COVID-19 was done in China, and it described comparable outcomes in both pregnant and nonpregnant adults with no vertical transmission [6]. However, subsequent studies were consistent with substantially increased maternal and neonatal morbidity and mortality risk in COVID-19-positive pregnant women [7]. Again, there are conflicting results about the vertical transmission of severe acute respiratory syndrome coronavirus 2 (SARS-CoV-2) to neonates, with some studies reporting as much as 13% positivity in newborns and others reporting no transmission at all [7-8]. The COVID-19 pandemic has reached multiple peaks of high case numbers (i.e., “waves”) around the world owing to its frequent mutations with variable effects on populations. There is a lack of comparison between COVID-19 cases of varying severity and perinatal outcomes in the international literature, especially for second wave cases. A study in Britain showed that pregnant women are more prone to develop a severe infection during the second wave [8].

Moreover, various laboratory and radiological parameters are scarcely studied in pregnant women in the third trimester who develop severe COVID-19. Therefore, the primary aim of this study was to assess the maternal-fetal outcomes of critically ill pregnant women diagnosed with COVID-19 pneumonia who required admission to the ICU. We also compared those outcomes with maternal-fetal outcomes of pregnant women with mild to moderate COVID-19. The secondary outcomes included characteristics of critically ill pregnant women, associated risk factors, comorbidities, mode of delivery, laboratory infection markers, and chest X-ray findings.

## Materials and methods

We conducted a retrospective observational study at Latifa Hospital, Dubai Health Authority [Dubai, United Arab Emirates (UAE)]. All procedures were conducted per the institutional ethical standards, and there was no interference in any treatment protocol. The total duration of the study was four months, and data were retrieved retrospectively from the hospital database and then prospectively extra-plotting it in a proforma. We included all booked or unbooked COVID-19-positive women [confirmed by reverse transcription (RT)-polymerase chain reaction (PCR)] aged 22-44 years and between 22 and 42 weeks of gestation from December 1, 2020, to March 31, 2021. We excluded patients younger than 22 years or older than 44 years and those in their first or second trimester. 

Patients were closely followed from admission to hospital discharge after the symptoms have completely resolved and the swab test was negative. We collected various demographic parameters, including age, body mass index (BMI), nationality, prior history of travel or contact with a COVID-19 patient, comorbidities, gravida, parity, and gestational age at the time of delivery.

We noted clinical signs and symptoms and chest X-ray findings, with the severity score assigned by the same consultant radiologist for all patients. All the patients did not receive prior COVID-19 vaccination and received the same standard treatment as per hospital protocol. The scoring system was semiquantitative, where each lung was divided into three zones and graded from 0 to 3 based on opacities in that zone [9]. Perinatal maternal-fetal outcomes were also recorded. The antenatal ultrasounds were also performed and no anomalies were detected. The fetal reverse transcriptase-polymerase chain reaction (RT-PCR) samples were obtained from the nasopharynx on the first-day postdelivery, and neonates were followed closely for signs and symptoms of respiratory distress for one week.

The data were analyzed using IBM SPSS Statistics for Windows, Version 26.0 (IBM Corp., Armonk, NY). The variables were compared between two groups using an independent t-test for parametric means, Whitney U test for nonparametric means, and Chi-square for percentages keeping p-values < 0.05 as significant.

## Results

One thousand one hundred eighty-four pregnant women reported to our hospital during their third trimester during the study period. Nasopharyngeal plus oropharyngeal swabs were taken for RT-PCR, and 123 (10.38%) were positive for COVID-19. Among the 123 positive patients, 93 cases (75.6%) experienced mild to moderate symptoms, and 30 patients (24.4%) experienced severe COVID-19 symptoms requiring ICU admission. The mean age of the study population was 32.6 ± 5.7 years; the mean BMI was 31.28 ± 5.8 kg/m2. Fifty-six patients (45.5%) were local UAE nationals, 21 (17.1%) were from other Middle Eastern countries, 26 (21.1%) patients belonged to the Indo-Pak subcontinent, and 20 (16.3%) had other diverse nationalities. Only 23 cases (18.7%) had a prior positive history of contact with COVID-19 patients or travel to an endemic area. The most common symptom was cough, present in 54 patients (43.9%), followed by fever in 49 patients (39.8%), shortness of breath in 35 patients (28.5%), and chest pain in 15 patients (12.2%). In comorbidities, gestational diabetes was present in 24 cases (19.5%), followed by obesity in 10 (8.1%), anemia in 10 (8.1%), hypertension in seven (5.7%), and three patients had asthma. All patients were nonsmokers. The demographic comparison between mild to moderate disease and severe cases is shown in Table 1.

**Table 1:** Demographic comparison between mild to moderate and severe COVID-19 infected pregnant women in their third trimester. COVID-19, coronavirus disease 2019; BMI, body mass index; UAE, United Arab Emirates; GDM, gestational diabetes mellitus; HTN, hypertension; SD, standard deviation

Demographic variable	Mild to moderate COVID-19 (n=93)	Severe COVID-19 (n=30)	p-value
Age in years, mean ± SD	31.7 ± 5.6 years	35.6 ± 5.0 years	0.001
BMI, kg/m^2 ^mean ± SD	30.968 ± 5.932	32.260 ± 5.735	0.298
Nationality			0.284
UAE (n)	46	10	
Arab (n)	13	8	
Sub-continent (n)	20	6	
Others (n)	14	6	
Gravida, mean ± SD	3.44 ± 2.329	3.07 ± 1.639	0.416
Parity, mean ± SD	2.01 ± 1.809	1.97 ± 1.474	0.904
Gestational age at admission in weeks, mean ± SD	36.58 ± 3.405	33.33 ± 2.928	< 0.001
Comorbidities			0.382
GDM (n)	16	8	
Obesity (n)	7	3	
Anemia (n)	7	3	
HTN (n)	6	1	
Asthma (n)	3	3	
Symptoms			
Cough (n)	26	28	< 0.001
Fever (n)	24	25	< 0.001
Dyspnea (n)	24	11	< 0.001
Chest pain (n)	6	9	0.004
Blood group			0.458
B positive (n)	26	9	
O positive (n)	32	6	
A positive (n)	23	12	
AB positive (n)	7	2	
Negative groups (n)	5	1	

The distribution of laboratory parameters is shown in Table 2. Three blood cultures were positive among severe COVID-19 patients, of which two were Staphylococcus aureus, and one was Pseudomonas. The maternal outcomes are shown in Table 3. A total of 132 babies were born to COVID-19-infected mothers, of which there were two twin pregnancies. The mean birth weight of all neonates was 2607.5 ± 700.5 g.

**Table 2:** Radiological and laboratory variable comparison between mild to moderate and severe COVID-19 infected pregnant women. COVID-19, coronavirus disease 2019; LDH, lactate dehydrogenase; ALT, alanine transferase; AST, aspartate aminotransferase; SD, standard deviation; CRP, C-reactive protein

Laboratory and radiological parameters	Mild to moderate COVID-19 (n=93)	Severe COVID-19 (n=30)	p-value
Chest X-ray severity score, mean ± SD	4.69 ± 2.880	11.43 ± 1.869	< 0.001
White blood count (x10^9^/L), mean ± SD	9.590 ± 3.825	12.723 ± 4.301	< 0.001
Platelet count (x10^9^/L), mean ± SD	203.9 ± 63.46	221.2 ± 150.4	0.372
Hemoglobin levels (g/dL), mean ± SD	11.066 ± 1.903	9.957 ± 1.322	0.004
CRP (mg/L), mean ± SD	24.138 ± 33.083	86.327 ± 69.192	< 0.001
Pro-calcitonin levels (ng/mL), mean ± SD	0.094 ± 0.232	0.668 ± 1.135	0.01
D-Dimer levels (µg/mL), mean ± SD	2.755 ± 3.469	2.346 ± 4.044	0.591
LDH levels (U/L), mean ± SD	170.1 ± 107.6	324.7 ± 161.7	< 0.001
Ferritin levels (µg/L), mean ± SD	93.66 ± 123.99	290.69 ± 328	< 0.001
ALT Levels (IU/L), mean ± SD	25.49 ± 31.35	47.27 ± 49.24	0.029
AST Levels (U/L), mean ± SD	29.88 ± 32.12	38.20 ± 27.57	0.174
Creatinine (mg/dL), mean ± SD	0.43 ± 0.127	0.43 ± 0.182	0.971
Potassium levels (mEq/L), mean ± SD	3.38 ± 1.02	3.790 ± 0.56	0.04
Blood cultures positivity, n (%)	-	3 (14.2%)	0.001

**Table 3:** Maternal outcome between mild to moderate and severe COVID-19 infected pregnant women. COVID-19, novel coronavirus disease 2019; PPH, postpartum hemorrhage; NVD, normal vaginal delivery; LSCS; lower segment Cesarean section; SD, standard deviation

Maternal outcomes	Mild to moderate COVID-19 (n=93)	Severe COVID-19 (n=30)	p-value
Mortality	-	6	< 0.001
Postpartum complications			< 0.001
Respiratory complications (n)	1	10	
PPH (n)	5	4	
Others (n)	3	1	
Indication of Cesarean			< 0.001
Fetal distress (n)	24	7	
Worsening COVID-19 (n)	13	18	
Other causes (n)	14	2	
Duration of hospital stay (days), mean ± SD	5.20 ± 6.457	12.33 ± 7.092	< 0.001
Mode of delivery			0.001
NVD (n)	55	6	
LSCS (n)	38	24	

There were two cases (1.6%) of vertical transmission in our study as COVID-19 RT-PCR was positive in neonates born to mothers with mild disease. The neonatal outcomes are elaborated in Table 4. Further risk assessment for mortality in severe COVID-19 cases is given in Table 5.

**Table 4:** Fetal outcomes between mild to moderate and severe COVID-19-positive pregnant women. COVID-19, novel coronavirus disease 2019; NICU, neonatal intensive care unit; SD, standard deviation.

Maternal outcomes	Mild to moderate COVID-19 (n=95)	Severe COVID-19 (n=30)	p-value
Birth weight (g), mean ± SD	2725.61 ± 714.14	2241.3 ± 512.7	0.001
Low birth eight (n)	13	14	0.001
Apgar score at birth, mean ± SD	8.94 ± 9.599	6.70 ± 1.179	0.03
Apgar score after 5 min, mean ± SD	8.97 ± 1.81	8.50 ± 0.861	0.176
Umbilical cord pH, mean ± SD	7.220 ±0.522	7.230 ± 0.079	0.917
Steroids administered prior to delivery (n)	23	20	< 0.001
Preterm delivery (n)	34	23	< 0.001
Stained liquor (n)	10	4	0.744
Fetal outcome (n)			0.341
Healthy (n)	84	26	
NICU admission (n)	7	4	
Death/Stillbirth (n)	4	-	

**Table 5:** Risk factor assessment of mortality among severe COVID-19 patients. COVID-19, coronavirus disease 2019; BMI, body mass index; UAE, United Arab Emirates; GDM, gestational diabetes mellitus; HTN, hypertension; ICU, intensive care unit; LDH, lactate dehydrogenase; ALT, alanine transferase; SD, standard deviation; CRP, C-reactive protein

Demographic variable	Severe COVID-19 patients who recovered (n=24)	Severe COVID-19 patients who died (n=6)	p-value
Age ≥ 30 years (n)	21	6	0.361
BMI ≥ 30 kg/m^2 ^(n)	15	4	0.298
Nationality			0.524
UAE (n)	9	1	
Arab (n)	5	4	
Sub-continent (n)	5	1	
Others (n)	5	1	
Gravida, mean ± SD	3.04 ± 1.706	3.17 ± 1.472	0.871
Parity, mean ± SD	1.92 ± 1.501	2.17 ± 1.472	0.717
Gestational age at admission (weeks), mean ± SD	33.92 ± 2.781	31 ± 2.449	0.026
Comorbidities			0.278
GDM (n)	7	1	
Obesity (n)	1	2	
Anemia (n)	3	-	
HTN (n)	3	-	
Asthma (n)	1	-	
Symptoms			
Cough (n)	22	6	0.464
Fever (n)	20	5	1
Dyspnea (n)	19	5	0.819
Chest Pain (n)	7	2	0.842
Duration of hospital stay (days), mean ± SD	10.29 ± 3.782	20.51 ± 11.22	0.012
Duration of ICU stay (days), mean ± SD	7.04 ± 3.282	14.83 ± 11.125	0.035
Ventilation assistance required (n)	9	6	0.008
Duration of intubation (days), mean ± SD	4.60 ± 2.221	10.17 ± 11.652	0.377
Chest X-ray severity score, mean ± SD	11.17 ± 1.659	12.5 ± 2.429	0.120
White blood count (x10^9^/L), mean ± SD	11.775 ± 3.678	16.51 ± 4.844	0.013
Platelet count (x10^9^/L), mean ± SD	235 ± 162.7	167 ± 70.7	0.332
Hemoglobin levels (g/dL), mean ± SD	10.32 ± 1.16	8.550 ± 0.965	0.002
CRP (mg/L), mean ± SD	76.22 ± 31.32	126.75 ± 144.23	0.678
Pro-calcitonin levels (ng/mL), mean ± SD	0.642 ± 1.091	0.770 ± 1.409	0.810
D-Dimer levels (µg/mL), mean ± SD	1.365 ± 1.127	6.27 ± 8.119	0.097
LDH levels (U/L), mean ± SD	294 ± 127.1	447.5 ± 234.1	0.035
Ferritin levels (µg/L), mean ± SD	268.5 ± 306.4	379.5 ± 424.7	0.468
ALT levels (IU/L), mean ± SD	39.7 ± 28.12	77.5 ± 95.4	0.407

## Discussion

To the best of our knowledge, our study is the largest conducted in the UAE that compares maternal-fetal outcomes in COVID-19 patients. A previous study in our hospital identified a total of seven pregnant patients with critical COVID-19 pneumonia admitted during the first wave of the pandemic [10]. During our study, 30 patients (24.3%) were admitted to the ICU, and 12 required invasive ventilation, meaning that the second wave was more deleterious for pregnant women. A systemic review evaluated an ICU admission rate of 9.6% among pregnant women, and most of those women were in their third trimester [1]. The higher rate in our study might be due to our study design, as only women in their third trimester were evaluated. In addition, our hospital was explicitly designated for the management of all COVID-19 cases in the region and received complicated cases. While the high rate in our study might be due to the emergence of a new viral strain, data do not yet exist to support this.

Severe COVID-19 was significantly associated with higher mortality (20% vs. 0%; p < 0.001), postpartum complications (50% vs. 9.67%; p < 0.001), and increased overall hospital stay (p < 0.001) than mild COVID-19. Similar studies reported higher rates of maternal mortality, morbidity, and early Cesarean section delivery primarily due to the mother's deteriorating health or fetal distress [11-13]. It was also evident in our study that neonates born to severe COVID-19 patients had significantly higher chances of being born preterm (76.6% vs. 35.7%; p < 0.001) and had low birth weight (46.6% vs. 13.9%; p = 0.002) than those born to mothers with milder COVID-19 disease. However, there were four cases of stillbirth in those with mild COVID-19, two cases of vertical transmission in mild cases, and no neonatal deaths, indicating that overall newborn outcomes are relatively better than outcomes for mothers. The above values are much higher than the average rate of stillbirth (4/1000 birth) and preterm births (6.1%) in the UAE [14]. Increased referrals can explain the higher mortality rate from periphery centers as three of the four stillbirths were diagnosed in community health units and transferred to this hospital for definitive management. A study by Schwartz showed better neonatal outcomes and no intrauterine spread of novel coronavirus [15]. On the contrary, numerous case reports and publications have confirmed vertical transmission in newborns, but the rate was very low [16].

The laboratory and radiological indices showed statistically significant higher mean chest X-ray score, total leukocyte count (TLC), and lower hemoglobin levels for severe cases. The levels of C-reactive protein (CRP), alanine transaminase, pro-calcitonin, lactate dehydrogenase, and ferritin were also significantly elevated in severe COVID-19 cases. The literature describes conflicting results, but most studies report that raised CRP and TLC were reliable indicators of severity in COVID-19 pregnant women [17-19]. The third trimester of pregnancy is considered a risk factor for severe COVID-19 [1, 8]. We found increasing age and symptoms of fever, cough, and dyspnea to be significantly associated with severe disease.

A subanalysis of mortality cases comparing severe COVID-19 with mild COVID-19 showed lower gestational age, increased duration of hospital stay and ICU admission, invasive ventilation, higher TLC, and lower hemoglobin were significantly associated with mortality in severe cases.

Our study was limited by its retrospective design. Additional workup was not possible, and treatment protocols were not studied, nor was amniotic sampling conducted for evidence of vertical transmission.

## Conclusions

Pregnant women with severe COVID-19 have high mortality, peripartum complications, increased hospital stay, and are more likely to undergo Cesarean section delivery because of COVID-19 progression. The neonates born to such mothers may be premature and have low birth weights. Increased age and presence of symptoms in pregnant women during their third trimester may be associated with the development of severe COVID-19. Therefore, healthcare professionals caring for symptomatic pregnant women who are relatively old should monitor these patients closely to improve overall outcomes.
